# Single-wall carbon nanohorns inhibited activation of microglia induced by lipopolysaccharide through blocking of Sirt3

**DOI:** 10.1186/1556-276X-8-100

**Published:** 2013-02-22

**Authors:** Lihong Li, Jinqian Zhang, Yang Yang, Qiang Wang, Li Gao, Yanlong Yang, Tao Chang, Xingye Zhang, Guoan Xiang, Yongmei Cao, Zujin Shi, Ming Zhao, Guodong Gao

**Affiliations:** 1 Department of Neurosurgery, Tangdu Hospital, Fourth Military Medical University, 710038, Xi’an, China; 2 Institute of Infectious Diseases, Beijing Ditan Hospital, Capital Medical University, 100015, Beijing, China; 3 Department of General Surgery, the Second People’s Hospital of Guangdong Province, 510515, Guangzhou, China; 4 International Mongolian Medical Hospital of Inner Mongolia, 010065, Hohhot, China; 5 Beijing National Laboratory for Molecular Sciences, State Key Laboratory of Rare Earth Materials Chemistry and Applications, College of Chemistry and Molecular Engineering, Peking University, 100871, Beijing, China; 6 Department of Chemical Biology, School of Pharmaceutical Sciences, Peking University, 100191, Beijing, China

**Keywords:** Single-walled carbon nanohorns, Septic encephalopathy, Cell proliferation, Apoptosis, Lipopolysaccharide, Sepsis, Sirt3

## Abstract

Single-wall carbon nanohorns (SWNHs) have been demonstrated to accumulate in cytotoxic levels within organs of various animal models and cell types, which emerge as a wide range of promising biomedical imaging. Septic encephalopathy (SE) is an early sign of sepsis and associated with an increased rate of morbidity and mortality. Microglia activation plays an important role in neuroinflammation, which contributes to neuronal damage. Inhibition of microglia activation may have therapeutic benefits, which can alleviate the progression of neurodegeneration. Therefore, we investigated the functional changes of mice microglia cell lines pre-treated with or without lipopolysaccharide (LPS) induced by SWNHs. To address this question, the research about direct role of SWNHs on the growth, proliferation, and apoptosis of microglia cell lines in mice (N9 and BV2) pre-treated with or without LPS had been performed. Our results indicate that the particle diameter of SWNHs in water is between 342 to 712 nm. The images in scanning electron microscope showed that SWNHs on polystyrene surface are individual particles. LPS induced activation of mice microglia, promoted its growth and proliferation, and inhibited its apoptosis. SWNHs inhibited proliferation, delayed mitotic entry, and promoted apoptosis of mice microglia cells. The effects followed gradually increasing cultured time and concentrations of SWNHs, especially in cells pre-treated with LPS. SWNHs induced a significantly increase in G1 phase and inhibition of S phase of mice microglia cells in a dose-manner dependent of SWNHs, especially in cells pre-treated with LPS. The transmission electron microscope images showed that individual spherical SWNH particles smaller than 100 nm in diameters were localized inside lysosomes of mice microglia cells. SWNHs inhibited mitotic entry, growth and proliferation of mice microglia cells, and promoted its apoptosis, especially in cells pre-treated with LPS. SWNHs inhibited expression of Sirt3 and energy metabolism related with Sirt3 in mice microglia cells in a dose-dependent manner, especially in cells pre-treated with LPS. The role of SWNHs on mice microglia was implicating Sirt3 and energy metabolism associated with it.

## Background

Sepsis-induced encephalopathy is caused by systemic inflammation in the absence of direct brain infection and clinically characterized by slowing of mental processes, impaired attention, disorientation, delirium, or coma. Importantly, septic encephalopathy (SE) is an early sign of sepsis and associated with an increased rate of morbidity and mortality. The pathogenesis of SE is unlikely to be directly induced by a pathogenic toxin, because similar encephalopathy can develop as a result of a number of systemic inflammatory response syndromes that lack an infectious etiology (e.g., acute pancreatitis and burns). Clinical and experimental data suggested that a number of factors including the local generation of pro-inflammatory cytokines and impaired cerebral microcirculation. The imbalance of neurotransmitters or the negative impacts of peripheral organ failure contribute to the development of SE [1-3].

Microglia, innate immune cells of the CNS, become activated in response to injury and appear to have important role in the defense against invading microbes and in wound repair [4]. Microglia, the resident immune cells of the central nervous system, are normally quiescent but become activated after infection or injury [5]. Because activated microglia can promote both damage and protection [5], their numbers require strict regulation, in part by ‘activation-induced cell death’ (AICD). In view of the key participation of microglia in neurological disorders [6], the knowledge of the molecular mechanism about AICD is important. However, under certain pathophysiological circumstances, microglia may also contribute to neuronal toxicity. For example, factors released from activated microglia can amplify inflammatory processes that contribute to neurodegeneration [7]. To harness and modulate the activity of microglia, it would be useful to be able to target biologically active compounds specifically to these powerful cells.

Since Iijima’s laboratory first synthesized single-walled carbon nanohorns (SWNHs) in 1999 [8], most of researchers have drawn their attention to theoretical and applicative fields relating to the material. With its tip-closed single-wall nanoscale cavum structure and advantages of high purity, uniform size, and ease of dispersion in solvents, SWNHs have been considered as a promising carrier for drug delivery system [9-14]. Nevertheless, interaction between unmodified SWNHs and cells has not been reported, although effects of modified SWNHs on HeLa and murine macrophage RAW 264.7 cells were shown recently [15,16]. More researches were focused on biological effects of fullerene, graphene, and carbon nanotubes (CNTs) modified with various bioactive groups on multiple type cells [17-38]; they revealed that carbon nanoparticles could be internalized in cells and react with subcellular organelles, such as endosome, mitochondria, lysosome, and nucleus [24-28,30]. Besides, an endocytic and a passive diffusion pathway for multi- and single-walled CNTs transmembrane process [27,28], and an oxidative stress pathway for cellular apoptosis induced by carbon nanoparticles, were proposed [39,40].

It is very important how SWNHs material reacts with the cells for evaluating its biological functions. Moreover, researches on the interactions between SWNHs and the cell lines will be helpful for examining the difference of cytotoxic effects of the material on the cells. So far, the role and functional mechanism of SWNHs material itself in the microglia cells are still unclear. Herein, to address this question, direct mechanisms of raw SWNHs on the growth, proliferation, and apoptosis of mice microglia cell lines were studied. The remarkable behavior of SWNHs in N9 and BV2 cells will be revelatory for further study on the interactive mechanisms in mice microglia cells with SWNHs and their possible applications in clinical treatment of SE or other neurodegenerative diseases associated with microglia.

## Methods

### Synthesis of single-wall carbon nanohorns by arc discharge in air

For the synthesis of SWNHs, we used pure graphite rods (Ø8 mm) as the electrodes. Direct current arc discharge was carried out in a water-cooled stainless steel chamber. The discharge between two electrodes was ignited in buffer gas with a pressure of 400 Torr and the current was held at 120 A. As the anode was consumed, the rods were kept at a constant distance from each other of about 1 mm by rotating the cathode. When the discharge ended, the soot generated was collected under ambient condition. In the arc discharge process, graphitic particles dropped to the bottom of the chamber, so we only collected the soot deposited on the inner and upper wall of the reaction chamber. Morphology analysis of the samples was carried out on JEOL JSM-7401 (JEOL Ltd., Tokyo, Japan) scanning electron microscope (SEM). The SEM was operated at 100 and 10 kV, respectively. Raman spectra were recorded from 1,000 to 2,000 cm^−1^ with a Jobin Yvon HR-800 spectrometer (Horiba Instruments, Tokyo, Japan) with an excitation wavelength of 633 nm. Thermogravimetric analysis was performed on a Q50TGA thermogravimetric analyzer (Thermal Analysis Inc., New Castle, DE, USA) from room temperature to 1,173 K at a rate of 10 K/min under an air flow of 30 ml/min [41].

### Preparation of SWNHs-coated dishes

Purified SWNHs were synthesized by the arc discharge method [41]. C, H, N analysis was carried out on Vario EL III Element Analyzer (Elementar Analysensysteme GmbH, Hanau, Germany). Other elemental contents were determined on a S4-Explorer X-ray fluorescence spectrometer (Bruker Corporation, Billerica, MA, USA) with 1 kW power and wavelength dispersion mode. The SWNHs had a purity of >95 wt.% and contained <5 wt.% amorphous carbon as the dominant impurity. To prepare the homogeneous SWNHs coating, a diluted solution of SWNHs in ultrapure water (produced from Milli-Q system, Millipro, Billerica, MA, USA) was dispersed. The aliquot (10 μg/ml) of the dispersed SWNHs was immediately spotted onto a 60-mm non-treated polystyrene dish (normal PS), which has a low adhesive surface for suspension culture in order to decrease the influence of the base material layer. The dishes were dried at 60°C for 3 h and sterilized by UV irradiation (DM-5; Daishin Co., Ltd., Osaka, Japan) for 16 h.

The following abbreviations have been used in this paper for the SWNHs-coated dishes: SWNHs-coated dishes, SWNHs10 (0.21 μg/cm^2^), SWNHs20 (0.42 μg/cm^2^), SWCNHs30 (0.64 μg/cm^2^), and SWNHs40 (0.85 μg/cm^2^).

SWNHs40 PS dishes with a bottom area of about 1 cm^2^ were prepared for SEM measurements and contact angle determinations. Uncoated PS dishes were used as control. After pre-treated by spraying gold on the films of samples, SEM measurements were carried out using a SIRION field emission scanning electronic microscope (FEI Corporation Ltd., Hillsboro, OR, USA) with accelerating voltage of 10.0 kV.

Contact angles of water droplets (volumes 2 to 5 μl) on SWNHs/PS and uncoated PS surfaces were determined on Dataphysics OCA20 Contact Angle Measuring System (Dataphysics, Filderatadt, Germany) at 293 K.

### Surface roughness and topography

The surface area and mesopore size of SWNHs were determined by ASAP 2010 V3.02 E surface area analyzer (Micromeritics Instrument Corp., Norcross, GA, USA) with BET method. The sample was pre-treated at 298.15 K under vacuum for half an hour. Adsorptive gas is N_2_ and saturation pressure is about 765 mm Hg. Temperature of analysis bath liquid N_2_ is 77.41 K. for 5 s. Particle density of SWNHs was determined on AccuPyc 1330 Pycnometer at 291.3 K. The particle density was estimated from the high-pressure He buoyancy effect. This effect was measured gravimetrically up to 30 Mpa by an electronic micro-balance and pressure transducers. The particle size of 10 μg/ml SWNHs aqueous suspension was determined on Zetasizer V 2.0 (Malvern Instrument Ltd., Worcestershire, UK) at 298.3 K.

A film with 0.83 μg/cm^2^ SWNHs/Ps was prepared for SEM and contact angle determination. The culture dish was cut, and the area of every film is about 1 cm^2^. For comparison, polystyrene films of same area without SWNHs were also prepared. SEM measurements were carried out on XL30 S-FEG scanning electronic microscopy (FEI Corporation Ltd) with accelerating voltage of 10.0KV. The samples were treated by spraying gold on films.

### Cell culture

Mice microglia cell lines N9 and BV2 were cultured in Dulbecco’s modified Eagle’s medium (DMEM) supplemented with 10% fetal bovine serum (FBS) (Gibco, Invitrogen, CA, USA) and 1% penicillin-streptomycin-neomycin (PSN) antibiotic mixture (Invitrogen) at 37°C in a humidified 5% CO_2_/95% air environment for 5 days. Lipopolysaccharide (LPS) from *Escherichia coli* serotype O111:B4 (Sigma-Aldrich, St. Louis, MO, USA) were used in this study. The cells were treated with 100 ng/ml LPS.

Cells were seeded onto 60-mm SWNHs-coated dishes and then were cultured in DMEM with FBS and PSN at 37°C in a humidified 5% CO_2_/95% air environment for 48 h treated with or without LPS at the same time. All results from BV-2 were similar to those from N9.

### Cell synchronization, BrdU labeling, and mitotic index

The cells were synchronized by double thymidine block. Briefly, cells were plated at 40% confluency and arrested with 2 mM thymidine. The cells were incubated in DMEM with FBS and PSN at 37°C in a humidified 5% CO_2_/95% air environment for 48 h, and after which were incubated with DNA-lipid mixture for 3 h, then the cells were washed twice and incubated in fresh medium for additional 5 h. Subsequently, cells were cultured in medium containing 2 mM thymidine and 2 μg/ml puromycin for the second arrest and drug selection. After 16 h incubation, the cells were released into the cell cycle by incubation in fresh medium at SWNHs-coated dishes for 48 h treated with or without LPS at the same time. Cells were collected or fixed at indicated time points and subjected to specific analyses.

BrdU labeling was used to evaluate DNA synthesis. After release from the second thymidine arrest at indicated time points, cells were cultured for 48 h in 12-well plate coated with SWNHs, then the cells were pulse labeled with BrdU (50 μM) for 30 min. After three washes of phosphate buffered solution (PBS), cells were fixed with 1 ml of Carnoy’s fixative (three parts methanol 1:1 part glacial acetic acid) at −20°C for 20 min, and followed by three washes of PBS. Subsequently, DNA was denatured by incubation of 2M HCl at 37°C for 60 min, followed by three washes in borate buffer (0.1 M borate buffer, pH 8.5). After incubation with the blocking buffer, cells were stained with anti-BrdU antibody (1:100; BD Biosciences, Franklin Lakes, NJ, USA) overnight at 4°C. After three washes of PBS, the cells were incubated with Texas Red-conjugated anti-mouse goat IgG for 30 min at real-time. After washes, the cells were mounted and BrdU positive cells were manually scored under immunofluorescence microscope.

Mitotic events were scored by time-lapse video microscopy and DNA staining. The cells were synchronized as described above and then cultured in SWNHs-coated for 48 h treated with or without LPS at the same time. Real-time images were captured every 10 min with Openlab software (PerkinElmer Inc., Waltham, MA, USA). Mitotic events of control, cells were scored by their morphological change (from flat to round-up). For each experiment, at least 800 cells were videotaped, tracked, and analyzed. Alternatively, nocodazole (100 ng/ml) was added into the medium and after release, the cells were collected, fixed, and stained with DNA dye (Hoechst 33258; Invitrogen, Carlsbad, CA, USA). Mitotic cells were scored by nuclear morphology and DNA condensation.

### Cell cycle analysis

The cells cultured in SWNHs-coated for 48 h treated with or without LPS at the same time were dissociated with trypsin, washed, and resuspended in PBS as a single-cell suspension after cultured 48 h. The cells were fixed in 70% ethanol overnight, stained with propidium iodide (25 μg/ml) (Sigma), and incubated for 30 min at 37°C with RNase A (20 μg/ml). The cells group treated with PBS was used as the controls. The cells were assessed by flow cytometer (Becton Dickinson, San Jose, CA, USA) and the results were analyzed with Modifit software. The DNA content of the cells was then evaluated by fluorescence-activated cell sorting with a FACSCalibur (BD Immunocytometry Systems).

### Cell growth and proliferation assay

Cell growth in SWNHs-coated dishes for 48 h treated with or without LPS at the same time was determined by the colorimetric tetrazolium derived sodium 3′-[1-(phenylaminocarbonyl)-3,4-tetrazolium]-*bis*(4-methoxy-6-nitro) benzene sulfonic acid hydrate (XTT) assay (Roche Applied Science, Mannheim, Germany), and DNA synthesis of the cells was assessed by the BrdU (bromodeoxyuridine) incorporation assay (Roche Applied Science). For the cell growth and proliferation assay, at 48 h after culture, the cells of each group were re-seeded in SWNHs-coated 96-well plates at a density of 0.3 to 1 × 10^4^ cells per well. After 48 h, XTT and incorporated BrdU were measured colorimetrically using a microtiter plate reader (Bio-Rad Corp., Hercules, CA, USA) at a wavelength of 450 nm [42].

### Cell viability assay

Cell viability was determined using a CCK-8 cell viability assay kit (DOJINDO Laboratories, Japan). All cells (5 × 10^3^ cells/well) were pre-treated with various methods as indicated and then incubated 16 h in a 96-well plate. A 10 μL of cell viability assay kit solution was added to each well of the plate. After incubation for 1 h at 37°C in the dark, absorbances were measured at 450 nm using a multi-well plate reader [43].

### Determination of apoptosis

Apoptotic cells treated with SWNHs were identified by fluorescence-activated cell sorting (FACS) using Annexin V-Fluos (Biolegend, San Diego, CA, USA) following the protocol of the manufacturer.

### TEM

Cells were seeded onto 60-mm SWNHs-coated and control dishes and then cultured in DMEM at 37°C in a humidified 5% CO_2_/95% air environment for 48 h, then collected and fixed with 3% glutaraldehyde. For transmission electron microscope (TEM), ultrathin cells slices of 100 nm thickness were cut using an ultramicrotome and mounted on grids. The slices were contrasted with aqueous solution of uranyl acetate and lead citrate and examined on JEM-1400 Transmission Electron Microscope (JEOL Ltd, Japan) with accelerating voltage of 80 kV.

### Cellular oxygen consumption assay

Steady state cell respiration in cells was measured in nonbuffered DMEM containing 5.5 mM glucose for cells with XF24 analyzer (Seahorse Bioscience, North Billerica, MA, USA) according to the manual.

### ATP production assay

Steady state cellular ATP levels were measured by using ATP bioluminescence assay kit CLS II in accordance with the protocol (Roche).

### NAD assay

Nicotinamide adenine dinucleotide (NAD) assay was performed as previously described [44-46]. Cells were extracted in 0.5 N HClO_4_, neutralized with 3 M KOH/125 mM gly-gly buffer (pH 7.4), and centrifuged at 10,000×*g* for 5 min. Supernatants were mixed with a reaction medium containing 0.1 mM 3-[4,5-dimethylthiazol-2-yl]-2,5-diphenyl-tetrazolium bromide (MTT), 0.9 mM phenazine methosulfate, 13 units/ml alcohol dehydrogenase, 100 mM nicotinamide, and 5.7% ethanol in 61 mM gly-gly buffer (pH 7.4). The A560 nm was determined immediately and after 10 min, and results were calibrated with NAD standards.

### Western blot analysis

Western blots were prepared as described [45]. Neuron cultures were lysed and collected in radioimmunoprecipitation assay buffer (cell signaling) with 1 mM PMSF on ice for 30 min. Cell lysates were centrifuged at 14,000×*g* for 10 min, and cell extracts were mixed with a 1:4 volume of SDS-PAGE loading buffer (10% β-mercaptoethanol, 10% glycerol, 4% SDS, 0.01% bromophenol blue, and 62.5 mM Tris–HCl, pH 6.8) and heated to 65°C for 15 min. Five samples were loaded on a 10% resolving SDS-polyacrylamide gel and transferred to polyvinyldifluoridine membranes. Membranes were incubated overnight at 4°C with rabbit polyclonal anti-Sirt3 (1:500; Abcam, Pak Shek Kok, New Territories, Hong Kong), rabbit polyclonal anti-acetyl-lysine (1:1,000; Biomol, Enzo Life Sciences, Inc., Farmingdale, NY, USA), P53 antibody (Santa Cruz Biotechnology Inc., Santa Cruz, CA, USA; 1:1,000 dilution), β-actin (Santa Cruz, 1:1,000), caspase 3, 7 (Cell Signaling Technology Inc., Danvers, MA, USA; 1:1,000), and then reacted with anti-rabbit or anti-goat secondary antibodies (1:10,000; Vector Laboratories, Burlingame, CA, USA). Immunoreactivity was detected with luminol reagent (GE, Munich, Germany).

### Statistics

Continuous normally distributed variables were represented graphically as mean ± standard deviation (SD). For statistical comparison of quantitative data between groups, analysis of variance (ANOVA) or *t* test was performed. To determine differences between groups not normally distributed, medians were compared using Kruskal-Wallis ANOVA. The *χ*^2^ test was used when necessary for qualitative data. The degree of association between variables was assessed using Spearman’s non-parametric correlation. All statistical analyses were carried out using SPSS software version 13.0 (SPSS Inc., Chicago, IL, USA). Probabilities of 0.05 or less were considered to be statistically significant.

## Results and discussion

### Characterization of SWNHs

The result of elemental composition determination of the SWNHs material used in this work is shown in Additional file 1: Table S1. The result showed that the material contained 95.3% of carbon. The content of each of the transition metals was less than 0.1%. The total metal content was about 0.25%. Due to catalyst-free preparation method of the material, its metal impurities are from the graphite raw material.

The adsorptive isotherm plot and BJH pore size distribution of SWNHs material are shown in Additional file 1: Figures S1 and S2. The result showed that BET surface area was 631.55m^2^/g, higher than that reported previously [47]. Single point total pore volume of pores (diameter less than 308.7 nm at *P*/*P*_0_ 0.994) was 1.57 cm^3^/g. The particle density was 1.0077 g/cm^3^ (RSD 0.91%). It implies the existence of many closed pores in SWNHs (see Additional file 1).

The measurement of SWNHs particle size distribution (Additional file 1: Figure S3) showed that it ranged from 342 to 712 nm in aqueous suspension. An individual SWNHs particle is a dahlia-like spherical aggregate of nanohorns with a diameter of 80 to 100 nm. Thus, our result showed that the particles were secondary aggregations of primary spherical SWNHs aggregates in aqueous suspension.

### SEM and contact angle measurements of SWNHs-coated dishes

SEM images (Additional file 1: Figure S4) showed that SWNHs were individual spherical particles with diameters of 60 to 100 nm on the PS surface. The comparison with the diameter of SWNHs aggregates in aqueous suspension was shown in above section. It meant that the structure of secondary SWNHs aggregates were disintegrated into individual primary aggregates of SWNHs on PS surface after evaporation of water in the suspension. It is conjectured that the disintegration is due to the stronger stacking interactions between the benzene ring on the surface of PS and SWNHs than that between SWNHs aggregates.

Because SWNHs particles were unstable coated on PS surface, partial SWNHs particles on PS surface diffused to water droplet and suspended by buoyancy of water. Then a new SWNHs/PS surface with less SWNHs particles than original SWNHs/PS surface was formed, as a result, the hydrophobicity of the surface was lowered and it resulted in decrease of the contact angle (Additional file 1: Figure S5).

### SWNHs inhibited mitotic entry of N9 cells, especially in pre-treated with LPS

To assure how the SWNHs affect cellular mitosis, we incorporated BrdU into the control. We found that the accumulation of mitotic N9 cells pre-treated with or without LPS were significantly delayed by SWNHs at every time point followed with the increasing concentrations of SWNHs (*P* < 0.01). The accumulation of mitotic N9 cells pre-treated with LPS (Figure 1B) was much more than that without LPS (Figure 1A).

**Figure 1:** **SWNHs inhibited mitotic entry of N9 cells, especially in pre-treated with LPS.** To assure how the SWNHs affect cellular mitosis, we incorporated BrdU into the control. We found that the accumulation of mitotic N9 cells pre-treated with or without LPS was significantly delayed by SWNHs at every time point followed with the increasing concentrations of SWNHs (*P* < 0.01), and the accumulation of mitotic N9 cells pre-treated with LPS (**B**) were much more than that without LPS (**A**). The mitotic entry of N9 cells pre-treated with LPS (**D**) was more than N9 cells (**C**). SWNHs inhibited mitotic entry of N9 cells pre-treated with or without LPS significantly at every time point followed with the increasing concentrations of SWNHs (*P* < 0.01). The mitotic entry inhibited by SWNHs in N9 cells pre-treated with LPS (**D**) was more significant than N9 cells (**C**). All data are represented as mean ± SEM.

The mitotic entry of N9 cells pre-treated with LPS (Figure 1D) was more than N9 cells (Figure 1C). SWNHs inhibited mitotic entry of N9 cells pre-treated with or without LPS significantly at every time point followed with the increasing concentrations of SWNHs (*P* <0.01). The mitotic entry inhibited by SWNHs in N9 cells pre-treated with LPS (Figure 1D) was more significant than N9 cells (Figure 1C).

### SWNHs inhibited growth and proliferation of N9 cells, especially in pre-treated with LPS

By XTT assays, we investigated the effect of SWNHs on cell growth and found that the growth of N9 cells pre-treated with LPS (Figure 2B) was much more significant than that in N9 cells (Figure 2A). The growth of cells was significantly inhibited by SWNHs at each time point in a dose-dependent manner (*P* < 0.001), especially in cells pre-treated with LPS (Figure 2B).

**Figure 2:** **SWNHs inhibited growth and proliferation of N9 cells, especially in pre-treated with LPS.** By XTT assays, we investigated the effect of SWNHs on cell growth and found that the growth of N9 cells pre-treated with LPS (**B**) was much more significantly than N9 cells (**A**). The growth of cells were significantly inhibited by SWNHs at each time point in a dose-dependent manner (*P* < 0.001), especially in cells pre-treated with LPS (**B**). Cell viability was evaluated by CCK-8 assay. The result showed that the proliferation of N9 cells pre-treated with LPS (**D**) was much more significantly than N9 cells (**C**). The proliferation of N9 cells treated with SWNHs was significantly inhibited at each time point in a time and dose-dependent manner (**C** and **D**). The effect induced by SWNHs on N9 cells pre-treated with LPS (**D**) was far more than that cells pre-treated without LPS (**B**). All data are represented as mean ± SEM.

Cell viability was evaluated by CCK-8 assay. The result showed that the proliferation of N9 cells pre-treated with LPS (Figure 2D) was much more significant than that in N9 cells (Figure 2C). The proliferation of N9 cells treated with SWNHs was significantly inhibited at each time point in a time- and dose-dependent manner (Figure 2C,D). The effect induced by SWNHs on N9 cells pre-treated with LPS (Figure 2D) was far more significant than that cells pre-treated without LPS (Figure 2B).

### SWNHs affected cell cycle of N9 cells, especially in pre-treated with LPS

The cell cycle of N9 cells was affected by SWNHs in a dose-dependent manner, especially in cells pre-treated with LPS (Figure 3B). Followed with the increasing concentrations of SWNHs, the ratio of the G1 phase increased and S phase decreased significantly in N9 cells pre-treated with LPS (*P* < 0.01). The ratio of G2 phase decreased in N9 cells and it decreased until SWNHs30 and increased abruptly at the concentration of SWNHs40 in N9 cells pre-treated with LPS (*P* > 0.05). The effect induced by SWNHs on N9 cells pre-treated with LPS was more significant than on N9 cells (Figure 3A).

**Figure 3:** **SWNHs affected cell cycle of N9 cells, especially in pre-treated with LPS.** Cell cycle of N9 cells was affected by SWNHs in a dose-dependent manner, especially in cells pre-treated with LPS (**B**). Followed with the increasing concentrations of SWNHs, the ratio of the G1 phase increased and S phase decreased significantly in N9 cells pre-treated with LPS (*P* < 0.01), the ratio of G2 phase decreased in N9 cells and it decreased until SWNHs30 and increased abruptly at the concentration of SWNHs40 in N9 cells pre-treated with LPS (*P* > 0.05). The effect induced by SWNHs on N9 cells pre-treated with LPS was more significant than on N9 cells. All data are represented as mean ± SEM.

### SWNHs promoted cell apoptosis of N9 cells, especially in pre-treated with LPS

After the cells had been cultured onto SWNHs-coated dishes for 48 h, the effect of SWNHs on cell apoptosis distribution was determined by flow cytometry. Apoptosis of N9 cells (Figure 4A) and N9 cells pre-treated with LPS (Figure 4B) was promoted with the increasing concentrations of SWNHs (*P* < 0.001). The effect on apoptosis induced by SWNHs on N9 cells pre-treated with LPS was more significant than N9 cells.

**Figure 4:** **SWNHs promoted cell apoptosis of N9 cells, especially in pre-treated with LPS.** After the cells had been cultured onto SWNHs-coated dishes for 48 h, the effect of SWNHs on cell apoptosis distribution was determined by flow cytometry. Apoptosis of N9 cells (**A**) and N9 cells pre-treated with LPS (**B**) was promoted with the increasing concentrations of SWNHs (*P* < 0.001). The effect on apoptosis induced by SWNHs on N9 cells pre-treated with LPS was more significant than N9 cells. All data are represented as mean ± SEM.

### The growth N9 cells affected by SWNHs, especially in pre-treated with LPS

The 3 × 10^5^ liver cells were seeded onto 60-mm SWNHs-coated dishes, and then all cells were countered after cultured for 48 h. The number of N9 cells pre-treated with LPS (Figure 5B) was more significant than N9 cells (Figure 5A). Followed with the increasing concentrations of SWNHs, the number of N9 cells was decreased significantly in a dose-dependent manner, especially in pre-treated with LPS (Figure 5B) (*P* < 0.01).

**Figure 5:** **The growth N9 cells affected by SWNHs, especially in pre-treated with LPS.** The 3 × 10^5^ liver cells were seeded onto 60-mm SWNHs-coated dishes, and then all cells were countered after cultured for 48 h. The number of N9 cells pre-treated with LPS was more significant than N9 cells (**A**). Followed with the increasing concentrations of SWNHs, the number of N9 cells decreased significantly in a dose-dependent manner, especially in pre-treated with LPS (**B**) (*P* < 0.01). All data are represented as mean ± SEM.

### TEM images of N9 cells treated with SWNHs

N9 cells were treated with SWNHs untreated with LPS as control (Figure 6A). The size of N9 cells pre-treated with LPS (Figure 6B) and their nucleus were larger than that in control. The apoptotic bodies were observed in cytoplasm. The size of lysosome and mitochondria in N9 cells pre-treated with LPS (Figure 6B) were larger than that in control (Figure 6A). A lot of secretory vesicles were observed outside of cells treated with SWNHs.

**Figure 6:** **TEM images of N9 cells treated with SWNHs.** (**A**) N9 cells treated with SWNHs untreated with LPS as control (×15,000 magnification). Scale bar represents 1 μm. (**B**) N9 cells cultured onto SWNHs-coated dishes (0.85 μg/cm^2^) for 48 h pre-treated with LPS (×15,000 magnification). Scale bar represents 1 μm. The size of N9 cells pre-treated with LPS and their nucleus were larger than that of control. The apoptotic bodies were observed in cytoplasm. The size of lysosome and mitochondria in N9 cells pre-treated with LPS (**B**) were larger than that of control (**A**). A lot of secretory vesicles could be observed outside of cells treated with SWNHs. All data are represented as mean ± SEM.

### The mitochondrial functions of N9 cells affected by SWNHs, especially in pre-treated with LPS

Intact cellular basal oxygen consumption rates (OCR) of N9 cells pre-treated with or without LPS induced by SWNHs were measured by Seahorse XF24 analyzer. The OCR of N9 cells pre-treated with LPS (Figure 7B) was more significant than that in N9 cells (Figure 7A). Followed with the increased concentrations of SWNHs, the OCR of N9 cells decreased significantly in a dose-dependent manner, especially in pre-treated with LPS (Figure 7B) (*P* < 0.01).

**Figure 7:** **The mitochondrial functions of N9 cells affected by SWNHs, especially in pre-treated with LPS.** Intact cellular basal OCR of N9 cells pre-treated with or without LPS induced by SWNHs measured by Seahorse XF24 analyzer. The OCR of N9 cells pre-treated with LPS (**B**) was more significant than N9 cells (**A**). Followed with the increasing concentrations of SWNHs, the OCR of N9 cells decreased significantly in a dose-dependent manner, especially in pre-treated with LPS (**B**) (*P* < 0.01). Steady state cellular ATP levels of N9 cells pre-treated with or without LPS induced by SWNHs were measured too. The steady state cellular alkaline phosphatase (APT) level of N9 cells pre-treated with LPS (**D**) was more significant than N9 cells (**C**). Followed with the increasing concentrations of SWNHs, the steady state cellular ATP level of N9 cells decreased significantly in a dose-dependent manner, especially in pre-treated with LPS (**D**) (*P* < 0.01). All data are represented as mean ± SEM.

Steady state cellular ATP levels of N9 cells pre-treated with or without LPS induced by SWNHs were measured too. The steady state cellular APT level of N9 cells pre-treated with LPS (Figure 7D) was more significant than that in N9 cells (Figure 7C). Followed with the increased concentrations of SWNHs, the steady state cellular ATP level of N9 cells was decreased significantly in a dose-dependent manner, especially in pre-treated with LPS (Figure 7D) (*P* < 0.01).

### The NAD levels of N9 cells affected by SWNHs, especially in pre-treated with LPS

NAD levels were measured in N9 cells pre-treated with or without LPS induced by SWNHs. NAD level of N9 cells pre-treated with LPS (Figure 8B) were more significant than in N9 cells (Figure 8A). Followed with the increased concentrations of SWNHs, the NAD level of N9 cells pre-treated with (Figure 8B) or without LPS (Figure 8A) was decreased significantly in a dose-dependent manner, especially in pre-treated with LPS (Figure 8D) (*P* < 0.01).

**Figure 8:** **NAD levels of N9 cells affected by SWNHs, especially in pre-treated with LPS.** NAD levels were measured in N9 cells pre-treated with or without LPS induced by SWNHs. NAD level of N9 cells pre-treated with LPS (**B**) were more significant than in N9 cells (**A**). Followed with the increasing concentrations of SWNHs, NAD level of N9 cells decreased significantly in a dose-dependent manner, especially in pre-treated with LPS (**B**) (*P* < 0.01). All data are represented as mean ± SEM.

### Key factors involved in apoptosis *in vivo*

The expression levels of Sirt3 in N9 cells pre-treated with LPS (Figure 9B) was much more than that in the control of N9 cells (Figure 9A). The increased expression levels of Sirt3 decreased followed with the increasing concentrations of SWNHs, which is especially significant in pre-treated with LPS (Figure 9B). The expression levels of activation cleavage of P53, caspase-3, and caspase-7 correlated with apoptosis increased followed with the increasing concentrations of SWNHs, especially in pre-treated with LPS (Figure 9B).

**Figure 9:** **Key factors involved in apoptosis *in vivo*.** The expression levels of Sirt3 in N9 cells pre-treated with LPS (**B**) was much more than control of N9 cells (**A**). The increased expression levels of Sirt3 decreased followed with the increasing concentrations of SWNHs, which is especially significant in pre-treated with LPS (**B**). The expression levels of activation cleavage of P53, caspase-3, and caspase-7 correlated to apoptosis increased followed with the increasing concentrations of SWNHs, which is especially significant in pre-treated with LPS (**B**).

Sepsis and its complications are the leading causes of mortality in intensive care units accounting for 10% to 50% of deaths. Up to 71% of septic patients develop potentially irreversible acute cerebral dysfunction. Sepsis-induced SE is the leading cause of death in septic patients. On one side, the brain is especially susceptible to damage during sepsis and on the other side the brain dysfunction may actively contribute to the pathogenesis of SE. The existence of reciprocal interactions between the immune and central nervous systems (CNS) makes the brain be one of the most vulnerable organs during sepsis. Furthermore, brain dysfunction can influence the function of the autonomic nervous system and neuroendocrine system, which accelerates the occurrence of SE [1-3]. Microglia is the resident immune cell in the brain tissue and is among the first to respond to brain injury. Microglia are rapidly activated and migrate to the affected sites of neuronal damage where they secrete both cytotoxic and cytotrophic immune mediators [48]. Microglial activation plays an important role in neuroinflammation and SE, which contributes to neuronal damage. Inhibition of microglial activation may have therapeutic benefits that can alleviate the progression of neurodegeneration and SE [7].

Our results indicated that LPS induced activation of microglia, promoted its growth and proliferation, and inhibited its apoptosis. The status was converted by SWNHs. Our result showed that in aqueous suspension, the particles were secondary aggregations of primary spherical SWNHs aggregates. In the present study, we prepared SWNHs-coated dishes with homogeneous thin or thick films by coating non-modified SWNHs on the surface of a commercially available non-treated polystyrene dish (normal PS). The main advantages of our research with SWNHs-coated dishes were as follows: (1) coating with non-modified SWNHs and without binder, (2) coating with gradual concentrations of SWNHs, (3) PS surface as individual particles of SWNHs and high transparency, and (4) no influence from the base substrate (normal PS as a base material has a proper adhesiveness for cells). Therefore, we can evaluate the natural properties of SWNHs films for cell responses. Thin films were promising materials because they have individual particles of SWNHs, which are known to largely influence cell functions.

The contact angle of water droplet on PS surface was 44.9° which was less than SWNHs/PS, 74.5°. The phenomena indicated higher surface hydrophobicity of SWNHs/PS than PS film. After a few minutes, contact angle of water droplet on SWNHs/PS surface decreased to 64.7° (Additional file 1: Figure S5). Because SWNHs particles were unstable covered on PS surface, SWNHs particles were suspended by buoyancy force of water. The image of SEM showed that distances between neighbor SWNHs particles were about 500 nm which was far less than the diameter of water droplet. Such a surface phenomena similar to lotus leaf effect can be observed (Additional file 1: Figure S4).

We found that LPS induced activation of microglia, promoted its growth and proliferation, and inhibited its apoptosis. SWNHs inhibited mitotic entry, growth and proliferation of mice microglia cells, and promoted its apoptosis, especially in activation microglia cells induced by LPS. The results of Ding et al. showed that at high dosages, carbon nanoparticles can seriously impact the cellular functions in maintenance, growth, and differentiation [49]. These different cellular behaviors cited above can be partially ascribed to the differences of properties for different carbon nanomaterials-surface area, pore structure, particle size, length, diameter and curvature, and partially ascribed to different cell types. Besides, the status of modification of carbon nanomaterials - modified with different functional groups or compounds, or not modified at all - will affect their biological functions on cells [50,51].

Apoptosis is an active process of cell death that both involves physiological and pathogenic processes. We observed the distended nuclei and scant cytoplasm, cell shrinkage, membrane blebbing, chromatin condensation, and apoptotic body in the cytoplasm of mice microglia, especially in cells pre-treated with SWNHs. The features of these phenomena were typical during the apoptotic process [52-54].

Our results showed that the roles of SWNHs on mice microglia cells were related to energy metabolism. Sirt3 was the only sirtuin implicated in extension of life span in human [55]. It has been shown Sirt3 involved with mitochondrial energy metabolism and biogenesis [56] and preservation of ATP biosynthetic capacity in the heart [57]. Sirt3 was shown to regulate the activity of acetyl-CoA synthetase 2 (AceCS2), an important mitochondrial enzyme involved in generating acetyl-CoA for the tricarboxylic acid (TCA) cycle. In these studies, Sirt3 knockout resulted in a marked decrease of basal ATP level *in vivo*[58]. Recent studies in cardiomyocytes demonstrated the protective role of Sirt3 from oxidative stress and hypertrophy [59,60]. Accordingly, the evidences above suggest that Sirt3 also has a pivotal role in protecting neurons from injury due to conditions that promote bioenergetic failure, such as excitotoxicity. Mitochondrial localization of Sirt3 plays a role in various mitochondrial functions, such as maintaining basal ATP level and regulating apoptosis. Sirt3 has been shown to regulate energy homeostasis [57].

Continuous supply of energy is crucial for the neuron survival due to the requirement for large amounts of energy for high metabolic processes coupled with an inability to store energy [61,62]. Therefore, the neurons are highly susceptible to insults that lead to energy depletion, such as oxidative stress, excitotoxicity, and DNA damage [63,64]. As a critical factor in energy metabolism for cell survival, NAD has drawn considerable interest. NAD is an essential molecule playing a pivotal role in energy metabolism, cellular redox reaction, and mitochondrial function. Recent studies have revealed that it is important for maintaining intracellular NAD in promoting cell survival in various types of diseases, including axonal degeneration, multiple sclerosis, cerebral ischemia, and cardiac hypertrophy [59,65-70]. Loss of NAD decreases the ability of NAD-dependent cell survival factors to carry out energy-dependent processes, leading to cell death. Our results coincide with those; the roles of SWNHs on mice microglia cells related to energy metabolism were associated with Sirt3.

Mitochondrial enzymes play central roles in anabolic growth, and acetylation may provide a key layer of regulation over mitochondrial metabolic pathways. As a major mitochondrial deacetylase, Sirt3 regulates the activity of enzymes to coordinate global shifts in cellular metabolism. Sirt3 promotes the function of the TCA cycle and the electron transport chain and reduces oxidative stress. Loss of Sirt3 triggers oxidative damage and metabolic reprogramming to support proliferation. Thus, Sirt3 is an intriguing example of how nutrient-sensitive, posttranslational regulation may provide integrated regulation of metabolic pathways to promote metabolic homeostasis in response to diverse nutrient signals. The expression levels of Sirt3 in mice microglia cells was increased as induced by LPS (Figure 9B). However, increased expression levels of Sirt3 were decreased followed with the increasing concentrations of SWNHs, which is especially significant in pre-treated with LPS (Figure 9B). The roles of SWNHS on mice microglia was implicating Sirt3 and energy metabolism associated with it.

P53 and SIRT3 regulated the apoptosis of various mammalian cells. Caspase-3 and caspase-7 are the key factors among cysteine proteases which are critical for apoptosis of eukaryotic cells. Our results showed that the expression levels of SIRT3 were decreased, and those of caspase-3 and caspase-7, as well as that of activation cleavage of P53 increased for mice microglia cells (Figure 9) in a dose-dependent manner with the increasing concentrations of SWNHs, which is especially significant in pre-treated with LPS (Figure 9B). These results also indicate that SWNHs promoted cell apoptosis. The phenomenon was associated with Sirt3 and energy metabolism was related to Sirt3.

SWNHs may be as a novel opportunity or method for the research on treatment of septic encephalopathy by inhibiting activation of microglia through blocking of Sirt3.

## Conclusions

SWNHs inhibited mitotic entry, growth and proliferation of mice microglia cells, and promoted its apoptosis, especially in cells pre-treated with LPS. SWNHs inhibited expression of Sirt3 and energy metabolism related with Sirt3 in mice microglia cells in a dose-dependent manner, especially in cells pre-treated with LPS.

## Abbreviations

AceCS2: Acetyl-CoA synthetase 2; AICD: Activation-induced cell death; BrdU: Bromodeoxyuridine; CNS: Central nervous system; CNTs: Carbon nanotubes; DMEM: Dulbecco’s modified Eagle’s medium; FACS: Fluorescence-activated cell sorting; FBS: Fetal bovine serum; LPS: Lipopolysaccharide; NAD: Nicotinamide adenine dinucleotide; PSN: Penicillin–streptomycin-neomycin; SD: Standard deviation; SE: Septic encephalopathy; SEM: Scanning electron microscope; SWNHs: Single-wall carbon nanohorns; TCA: Tricarboxylic acid

## Competing interests

All authors declare that they have no competing interests.

## Authors’ contributions

LL, JZ, YY, QW, YC, ZS, MZ, and GG have carried out the molecular genetic studies, participated in the sequence alignment, and drafted the manuscript. LL, JZ, LG, YY, TC, XZ, GX, and GG participated in the design of the study and performed the statistical analysis. JZ and GG conceived of the study, and participated in its design and coordination and helped to draft the manuscript. All authors read and approved the final manuscript.

## Supplementary Material

Additional file 1 **Supporting Informations.** This file contain descriptions of the elemental contents of SWNHs material, adsorptive isotherm plot and BJH pore size distribution of SWNHs material, particle density of SWNHs, particle sizes distribution of SWNHs in aqueous suspension and the films of SWNHs/PS observed by SEM, and contact angle of water droplet on the surfaces of PS and PS coated with SWNHs(SWNHs/PS) films. Click here for file
